The article "FOXD1 Regulates the Sensitivity of Cetuximab by Regulating the Expression of EGFR in Head and Neck Squamous Cell Cancer" was retracted in 2023. Reasons: unreliable results or conclusions; concerns about the data; concerns about the results or conclusions; concerns about the peer review.

# FOXD1 Regulates the Sensitivity of Cetuximab by Regulating the Expression of EGFR in Head and Neck Squamous Cell Cancer

**DOI:** 10.1155/2022/6108241

**Published:** 2022-01-25

**Authors:** Lan Mu, Jian Zhang, Zhuo Wu, Jingxi Huang, Ying Cui

**Affiliations:** ^1^Department of Otorhinolaryngology Head and Neck Surgery, First Affiliated Hospital of Jinzhou Medical University, Jinzhou 121000, China; ^2^Communist Youth League Committee, First Affiliated Hospital of Jinzhou Medical University, Jinzhou 121000, China; ^3^Department of Gastroenterology, First Affiliated Hospital of Jinzhou Medical University, Jinzhou 121000, China

## Abstract

**Objectives:**

Previous experiments have shown that growth factor receptors play important role in tumor proliferation, metastasis, and therapeutic effect of chemotherapeutic drugs. At the same time, forkhead box D1 (FOXD1) plays an important role in a variety of signal transmission, but its expression profile was known little about head and neck cancer. The purpose of this experiment was to explore the regulation of FOXD1 on the tumor progression of head and neck cancer and to explore the correlation of FOXD1 on the expression of growth factor receptors (EGFR).

**Methods:**

The bioinformatics online database analyzed the expression of FOXD1 and EGFR in tumor tissues and nontumor tissues. Real-time quantitative PCR was used to detect the FOXD1 and EGFR expression in 45 tumor tissues and 15 nontumor tissues. The plasmid was used to construct FOXD1 overexpressing head and neck squamous cell cancer lines and observe the clonal formation and invasion of tumor cells under the intervention of EGFR-specific antibody—cetuximab.

**Results:**

The expression of FOXD1 and EGFR in tumor tissues was higher than that in nontumor tissues. The higher expression of FOXD1 and EGFR was not conducive to the prognosis of patients. The expression of FOXD1 and EGFR was positively correlated, and immunohistochemical analysis showed the high expression of FOXD1 and EGFR has close relation to the advanced stage of the tumor. In vitro cell experiments proved that overexpression of FOXD1 can partially offset the cloning ability of cetuximab on head and neck tumor cells.

**Conclusion:**

FOXD1 has an important regulatory role in the progression of head and neck cancer, and its abnormally high expression was not conducive to the prognosis of cancer patients. FOXD1 can regulate the expression of growth factor receptors in head and neck cancer, which provides a new idea for the better use of tumor growth factor receptor-specific antibodies for collaborative therapy.

## 1. Introduction

Head and neck cancer has a high mortality rate, usually as high as 50–80% within 24 months after diagnosis [1]. The patient's quality of life is severely impaired, usually accompanied by disturbances in swallowing, daily speech, chewing, and facial expressions [2]. Therapies currently approved by the FDA for the treatment of advanced metastatic head and neck cancer include cetuximab, an antibody that blocks the receptor tyrosine kinase (RTK) epithelial growth factor receptor (EGFR), and it is usually combined with other radiotherapy drugs for the treatment of advanced locally metastatic head and neck cancer [3, 4]. Although cetuximab can significantly prolong the median overall survival of head and neck cancer patients, the clinical remission rate was limited to late local disease with a course of about 10 months or metastatic disease with a course of 2-3 months [5–8]. Head and neck cancer patients were resistant to cetuximab since they received cetuximab, while a latest clinical study on patients receiving cetuximab monotherapy found that 87% of head and neck cancer patients had resistance to cetuximab since they received cetuximab, while the remaining 13% of patients responded to cetuximab sensitively at the beginning, but it has acquired drug resistance with the extension of the clinical application time of the drug. Therefore, it is urgent to clinically identify cetuximab sensitivity and the mechanism of cetuximab resistance in head and neck cancer because these results can effectively improve the therapeutic effect of cetuximab [9–11].

Transcription factors (TFs) participate in a wide range of biological functions as essential regulatory protein factors due to their powerful functions. Their dysfunction was closely related to many major diseases [12]. The forkhead box (FOX) family, composed of proteins that share related winged helix-turn-helix DNA binding motifs, belongs to the “winged helix” superfamily [13]. FOX genes are widely present in the evolution of vertebrates and invertebrates, involved in many molecular cascades and regulation of biological functions, such as embryonic development, cell cycle regulation, early morning metabolism control, and signal pathway transduction [14]. FOXD1 dysfunction has been linked to different pathologies, which constitutes diagnostic biomarker and becomes a promising target for future treatment [14].

In this study, we were surprised to find that FOXD1 has abnormally high expression in head and neck cancers. Data analysis and experiments have shown us that FOXD1 can regulate EGFR expression. For head and neck cancers with high EGFR expression at the same time, this discovery can reveal the mechanism of cetuximab resistance in patients with head and neck cancer and the clinical application of new therapeutic targets was of great significance.

## 2. Materials and Methods

A total number of 45 patients with head and neck cancer were treating in First Affiliated Hospital of Jinzhou Medical University from 2015 to 2020. All patients signed a preinformed consent, and the study was approved by our institutional review board. The patients were selected without any history of radiotherapy surgery, or chemotherapy; the archived tissues were stained according to established histopathological standards to determine the previous test results. At the same time, 15 healthy paracancer tissues were obtained and professionally identified by experienced pathologists.

### 2.1. The Immunohistochemical Staining

4M sections were prepared. After dewaxed with xylene, ethanol was graded and treated with citric acid buffer (pH 6.0) followed by microwave antigen treatment for 15 minutes. The activity of endogenous peroxidase was blocked by hydrogen peroxide, and histochemical staining was performed by SP immunoassay. Diluted primary antibody (anti-FOXD1 polyclonal antibody) 1 : 200 Abcam, USA) was added, while the primary antibody group was replaced with PBS as the negative control. After the addition of secondary antibody for 20 min, rinse thoroughly with PBS, DAB color development, hematoxylin eosin staining, and put under the microscope after dehydration treatment.

### 2.2. Western Blot

Western blot according to the description of the operating instructions was provided by the manufacturer. Lysis buffer was used to lyse the cells. Bradford assay measures total cellular protein (BioRad, Hercules, calcium, USA). Equivalent protein lysates (20 g per pore) were electrophoreted in 10% sodium dodecyl sulfonate gel and then transferred to a polyethylenediene difluoride film (PVDF) (Bio-RAD, Richmond, CA, USA). 5% bovine serum was incubated for 1 hour, and then FOXD1 and EGFR-specific primary antibody were added and incubated at 4°C overnight. Anti-GAPDH was used as endogenous internal reference (all antibodies were from Santa Cruz Biotechnology, USA; all dilutions were 1 :  1000). After washing with PBS, add goat anti-rabbit. The protein bands were observed by using chemiluminescence detection system (ECL, Thermo Scientific, America).

### 2.3. Quantitative Real-Time Polymerase Chain

ReactionTrizol reagent (hot Fisher Scientific) was used to separate total RNA in a cell. The concentration and purity of RNA were tested by using a NanoDrop2000 spectrophotometer (Thermo Scientific, Waltham, MA). Reverse transcriptase kit was used to reverse transcribe RNA into cDNA according to the operating requirements of the instructions. The specific setting parameters of polymerase chain reaction (PCR) were reaction at 95°C for 3 minutes, reaction at 95°C for 3 minutes for 40 cycles, and reaction at 58°C for 30 s. GAPDH serves as an endogenous standard reference to which all results are unified. The priming sequence is FOXD1 (sense: 5′-ActGGCTTACatTTCCGTCAAC-3′, antisense: 5′-gTTcTTTttgtcatagatgtccgtg-3′) and GAPDH (forward: 5′-GGGAGCCAAAAGGGTcat-3′ and reverse: 5′-gagTCCTTCCACGATACCAA-3′). All RT-QPCR data were calculated and represented using 2^−△△ct^ and then converted to fold changes.

### 2.4. Colony Formation Assay

Cells were transfected with PCDNA 3.1-FOXD1 or pcDNA-NC, and cell suspension (1 × 10^3^ cells per well) was plated at 0.5% agarose-coated 6-well plates and treated with carboplatin (15.0 *μ*g/ml) for 48 h. In fortnight, cells were washed and fixed with 10% formaldehyde and then stained with crystal violet and photographed.

### 2.5. Cell Invasion

The invasion test was carried out in a 24-well chemotactic cavity containing a fibrous pore membrane of 8 microns with matrix glue. In the upper compartment, about 2 × 10^4^ cells were added, with serum-free medium, and then medium containing 20% FBS was added to the lower compartment. The fiber membrane was obtained after 24 h of cell culture in a cell incubator. After methanol fixation, the excess attached cells were wiped with a cotton swab. After washed by PBS three times, the cells were stained by crystal violet. The degree of migration was represented by the average number of cells in 5 fields of vision.

### 2.6. Cell Culture

The Tu167 and LN212 cell lines were purchased from Tongpai (Shanghai) Biological Technology Co., Ltd. (Shanghai, China). Cells were cultured at 37°C in a humidified incubator with 5% CO_2_ in DMEM supplemented with 10% FBS, 100 U/mL penicillin, and 100 *μ*g/mL streptomycin.

### 2.7. pcDNA3.1-FOXD1-GFP

The overexpressed plasmid of FOXD1 (PCDNA3.1-FOXD1-GFP) and no-load plasmid (PCDNA3.1-NC) was transfected into head and neck cancer cell lines with Lipo2000 transfection reagent to constructed FOXD1 group and negative control group. The plasmid transfected positive clones were screened with puromycin (2 ug/ml) and amplified. The expression of FOXD1 at mRNA and protein levels after transfection was detected by real-time PCR and Western blot. After that, the FOXD1 group and negative control group were treated with or without cetuximab 12.5 *μ*g/Ml.

### 2.8. Statistical Analysis

SPSS 17.0 software was used for statistical analysis of the experimental data. Groups of data are represented by mean ± SD (standard deviation). Independent sample *T*-test was used for the comparison of mean values between the two groups. *P* < 0.05 was considered statistically significant.

## 3. Results

### 3.1. Abnormally High Expression of FOXD1 and EGFR in Head and Neck Cancer

Through bioinformatics search, the expression of FOXD1 in tumor tissues is significantly higher than that in nontumor tissues (Figure 1(a)). Similarly, by searching for the expression of EGFR in salivary glands and head and neck cancer tissues, we can unambiguously find that EGFR was basically not expressed in salivary glands thyroid and tongue muscles, but there were extremely high expression levels in immunohistochemical sections in tumor tissues (Figure 1(b)). Next, in order to further verify the above conclusions, QRTPCR analyzed the mRNA levels of FOXD1 and EGFR in 45 tumors and 15 nontumor tissues (Figures 1(c) and 1(d)). From the experimental results, it can be clearly found that the expression levels of FOXD1 and EGFR in tumor tissues are higher than those in nontumor tissues. These experimental results can fully explain the high expression of FOXD1 and EGFR in head and neck cancer.

The expression levels of FOXD1 and EGFR are closely related to the life cycle of patients.

In order to further understand the impact of FOXD1 and EGFR expression levels on the survival of patients with head and neck cancer, we were surprised to find that FOXD1 plays an important role in the life cycle of tumor patients through the analysis of the online bioinformatics database. As shown in the Figures 2(a) and 2(b), the overall survival and disease-free survival of patients with low FOXD1 expression was significantly higher than that in the high expression group. At the same time, we analyzed the impact of EGFR on patient survival and found that the high expression of EGFR has an adverse effect on the survival of patients with head and neck cancer (Figure 2(c)). Patients with high EGFR expression have a lower survival time compared with patients with low EGFR expression. Through immunohistochemical analysis (Figure 2(d)), we can clearly find that the expression levels of FOXD1 and EGFR in the T3 stage of advanced tumor tissues are higher than the expression levels of early T1. Through the above analysis, we can clearly draw the following conclusions: the expression levels of FOXD1 and EGFR have a very important impact on the survival of patients with head and neck cancer, and abnormally high expression is not conducive to the prognosis of patients.

There was a positive correlation between the level of FOXD1 and the level of EGFR in head and neck cancer.

In order to further understand the interaction and regulation of FOXD1 and EGFR, we were surprised to find that there was a close relationship between FOXD1 and EGFR through bioinformatics data analysis. The expression levels of FOXD1 and EGFR are positively correlated in the pathological tissues of head and neck cancer (Figure 3(a)). In order to make the above conclusion clearer, we analyzed the relationship between the two at the mRNA level by real-time quantitative PCR.  Figure 3(b) shows that FOXD1 and EGFR are positively correlated at the mRNA level. In order to further understand the specific regulation mode of FOXD1 and EGFR, we observe the effect on the expression level of EGFR through the high expression of FOXD1-specific expression plasmid. WB found that the overexpression of FOXD1 caused high expression of EGFR regardless of the level of mRNA or protein (Figures 3(c) and 3(d)). From this, we can conclude that FOXD1 can regulate the expression level of EGFR in patients with head and neck cancer.

High expression of FOXD1 can partially relieve the tumor suppressive effect of cetuximab on head and neck cancer cell lines.

Cetuximab is a clinically specific drug that is specifically used to treat tumor growth caused by high EGFR expression. In order to study the effect of FOXD1 on the antitumor effect of cetuximab, we established a specific in vitro FOXD1 overexpression cell line to achieve FOXD1 specificity high expression. Transwell clearly finds that the cell invasion ability of cells overexpressing FOXD1 was significantly increased compared with that of the control group, and the cell invasion ability was significantly decreased after the cells are treated with cetuximab alone. At the same time, we noticed that although the cells overexpression FOXD1 were treated with drugs, and the cell invasion ability was similar to that of the negative control group (Figure 4(a)). Subsequent cell clone formation experiments also obtained similar experimental results. From the results in Figure 4, it can be seen that the number of cell clones formed after FOXD1 overexpression was significantly increased compared with the NC group, and the number of cell clones after treatment with cetuximab was significantly reduced, while the inhibitory effect of cetuximab on cell clone formation in the FOXD1 overexpression cell line was significantly reduced, which was significantly different from the number of cell clone formation in the drug-only treatment group (Figure 4(b)). From this, we can know that FOXD1 has important regulatory significance for regulating the biological effects of cetuximab.

## 4. Discussion

EGFR (also called ERBB1/HER1) is a RTK belonging to the ERBB family. Cetuximab and panitumumab can bind to the extracellular domain of EGFR, thereby blocking receptor tyrosine kinases and various downstream signal transduction cascades related to cell proliferation, invasion, metastasis, and survival and angiogenesis reaction [15, 16]. A variety of signal transduction pathways are involved in the downstream biological effects activated by EGFR, such as RAS-RAF-MAPK, PI3K-PTEN-AKT, and JAK/STAT. Most of the above signal pathways are also involved in antibody-mediated resistance to EGFR inhibition machine [17–21]. Any gene changes in the signaling pathway, such as KRAS, NRAS, BRAF, and PIK3CA gene mutations, may lead to the constitutive activation of EGFR and subsequent changes in intracellular signaling to eventually achieve drug resistance [22, 23]. This has caused huge restrictions on the clinical application of cetuximab or head and neck cancer patients with advanced local or metastatic disease, and the clinical treatment standard is cetuximab combined with radiotherapy or chemotherapy, but in most cases, patients do not respond or are resistant to cetuximab treatment [24]. Unlike colorectal cancer and colorectal cancer, there is currently no clear and effective biomarker target for effective combination therapy in head and neck cancer [25]. By exploring the molecular mechanism of head and neck cancer resistance to cetuximab, it can promote the research progress of such biomarkers. Therefore, the discovery of specific drug resistance molecular mechanisms and regulatory signal pathways is beneficial to cetuximab and other groups that block receptor tyrosine kinases.

In our research, we found that FOXD1 is a new regulator of EGFR expression. FOXD1 was related to the occurrence and progression of a variety of tumors. Abnormal FOXD1 expression is involved in the progression of tumors including colorectal cancer [26], melanoma, breast cancer [27], glioma [28], osteosarcoma, renal cell carcinoma, medulloblastoma ovarian carcinoma, [29], and lung cancer [30]. However, the function of FOXD1 in head and neck tumor formation is poorly understood. In this study, we confirmed that FOXD1 was highly expressed in head and neck squamous cell cancer. Through bioinformatics analysis, we found that the expression level of FOXD1 and EFGR showed a positive correlation trend in patients with head and neck cancer. Subsequently, in order to verify the above results in specific experiments, we analyzed the correlation between the expression of ROXD1 and EFGR at the mRNA level in the collected 45 cases of tumor tissues. We are surprised to find that the experimental results obtained are consistent with the results obtained by bioinformatics analysis, so we judge that there must be an important regulation method between the FOXD1and EGFR. The next experiment is intended to prove the regulation between FOXD1 and EGFR. After overexpression of FOXD1, we found that, at the same time, the expression of EGFR was also significantly upregulated. By observing tumor tissue sections, we found that the immunohistochemistry of FOXD1 and EGFR staining is always performed simultaneously. When there is strong FOXD1 and EGFR staining in advanced tumor tissues, there is weak FOXD1 and EGFR staining in early tumor tissues. Since there are a large number of patients with head and neck cancer who are resistant to cetuximab, we wondered whether it was related to the abnormally high expression of FOXD1 in the tumor, so we established a cell line that overexpressed FOXD1 and passed cetuximab treatment of drugs. We found that, in cell lines with high FOXD1 expression, the clone formation and invasion ability of cells was improved compared with the non-high expression group. This means that the cells with high FOXD1 expression are less sensitive to cetuximab and have a certain degree of drug resistance, which reduces the antitumor effect of cetuximab. Therefore, we conclude that FOXD1 is likely to be an upstream regulator that regulates the expression of EGFR and plays an important role in the treatment of head and neck cancer with cetuximab. Abnormal expression of FOXD1 may be responsible for the production of cetuximab resistance. It should also be pointed out that our research needs to be further deepened to reveal the regulatory mechanism between FOXD1 and EGFR.

## Figures and Tables

**Figure 1:** Abnormal expression of FOXD1 and EGFR in HNSCC tissues (a). The mRNA levels of FOXD1 in tumor tissues and nontumor tissue (downloaded from GEPIA). (b) Representative immunohistochemical images of EGFR from salivary glands (1), thyroid (2), tongue muscle (3), and head and neck cancer tissues (4) (downloaded from the human protein Atlas http://www.proteinatlas.org/). The mRNA levels of FOXD1 (c) and EGFR (d) in 45 cases of HNSCC and 15 normal tissues.

**Figure 2:** Effects of FOXD1 and EGFR on prognostic survival in patients with HNSC. Effects of FOXD1 on overall survival (a) and disease-free survival (b) in patients with HNSCC. (c) Effects of EGFR on overall survival in patients with HNSC. (d) Representative images of FOXD1 and EGRF immunohistochemical staining at T3 and T1 stages of TNM staging.

**Figure 3:** There is a positive correlation between FOXD1 and EGFR. (a) The correlation between FOXD1 and EGFR is downloaded from A. (b) Correlation between FOXD1 and EGFR in 45 patients with head and neck cancer. (c) The effect of overexpressed FOXD1 on EGFR expression was detected by Westen blot. (d) The effect of overexpressed FOXD1 on EGFR expression was detected by RT-PCR.

**Figure 4:** Overexpression of FOXD1 can reverse the inhibitory effect of cetuximab on HNSCC cells. (a) Effects of FOXD1 overexpression on the invasion of HNSCC cells treated with cetuximab. (b) Effects of FOXD1 overexpression on the clonal formation of HNSCC cell lines treated with cetuximab.

## Data Availability

Data to support the findings of this study are available on reasonable request from the corresponding author.
